# Decision-Making Application of the Cloud-Fog Hybrid Model Based on the Improved Convolutional Neural Network in Financial Services in Smart Medical Care

**DOI:** 10.1155/2022/5732379

**Published:** 2022-08-09

**Authors:** Shan Lu

**Affiliations:** University of International Business and Economics, Beijing 100050, China

## Abstract

In order to alleviate the “difficulty in seeing a doctor” for the masses, continuously optimize the service process, and explore new financial service processes for admission and discharge, this study proposes a cloud-fog hybrid model UCNN-BN based on an improved convolutional neural network and applies it to financial services in smart medical care. Decision-making applications: this research improves and designs the UCNN network based on AlexNet and introduces small convolution layers to form convolution groups, making the network more adjustable. The network structure is simpler and more flexible, and it is easy to adjust the algorithm. The number of parameters is small, and it can be directly superimposed without having to add new network hidden layers. The experimental results show that the recognition rate of the UCNN network on the FER2013 and CK+ datasets is higher than that of other recognition methods, and the recognition rates on the FER2013 and CK+ datasets are 98% and 68.01%, due to other methods. This shows that the improved convolutional neural network used in this study for financial services in smart medical care has certain applicability, and small convolution kernels help to extract more subtle features, so as to identify more accurately.

## 1. Introduction

In the 1990s, two scholars, Michael Hammer and Jame Champy, put forward the theory of “business process reengineering” [1]. The core of which is to use advanced information technology and modern management methods to reengineer business processes to improve service quality and efficiency. Business goals [2]: the First Affiliated Hospital of Wenzhou Medical University applies the concept of “smart medical care” to the reconstruction of the financial service process of admission and discharge. With the help of information technology, a new model of financial service for admission and discharge is constructed, and the financial procedures for admission and discharge are directly handled by the nursing staff in the ward. Through the new model, the financial procedures for admission and discharge have been optimized, the waiting time of patients in line has been shortened, hospital costs have been reduced, and patient satisfaction has been significantly improved [3]. Smart healthcare consists of three parts, namely, the smart hospital system, the regional health system, and the family health system. The smart hospital system consists of a digital hospital and an improved application. The regional health system consists of a regional health platform and a public health system. The home health system is the health protection closest to the citizens, including those who cannot be sent to the hospital for mobility problems.The home medical system is suitable for chronic diseases, remote care of elderly and young patients, health monitoring of mentally retarded, disabled, infectious diseases and other special groups, and video medical treatment for patients. Its intelligent medication system can automatically prompt medication time, contraindications, remaining medication, etc.The financial part of this study belongs to the family health system.

Computing technology is already a very mature technology in today's computer market, and cloud computing service products produced by using cloud computing also play an important role in today's markets in various fields. There are many large, medium, and small enterprises in various fields using cloud computing products. Cloud computing can provide enterprises with functions such as information storage, management, and maintenance [4] and can also simplify the investment of enterprises in building networks, software, and systems. Human resources and the number of customers using cloud computing technology products are increasing, and it has been expanding from enterprise customers to individual users. Also, because of the increasing market demand, more and more information technology companies are moving their research centers to cloud computing technology research and product development. Major domestic and foreign information companies, including communication companies, are making efforts in this regard. Some researchers [5, 6] described the application of fog computing in IoT systems and its application characteristics; Pang et al. [5] placed computing at the edge of the cloud computing network to improve the availability and scalability of the system architecture and reduce transmission load and cloud processing burden. Rabinovich et al. [7] and Vaquero and Rodero-Merino [8] studied key technologies such as sensor network, peer-to-peer network, network virtualization in cloud-fog hybrid computing, and the main challenges faced by cloud-fog fusion. Zao et al. [9] studied the multilayer cloud and fog computing infrastructure and linked data network and its possible future intelligent environment in terms of the wearable user interface. Zhu et al. [10] studied the data access and interaction mechanism of edge network edge devices in fog computing. Giordano et al. [11] studied the layered distributed architecture of fog computing and its resource advantages in large-scale distributed computing based on the big data interference problem brought by the Internet of Things. Cloud computing is becoming an important force for change, but due to the proliferation of access devices and limited network bandwidth, the combination of fog computing or cloud-fog computing may bring about real computing changes.

A convolutional neural network is a method that can automatically extract object features, and feature extraction and feature classification are a simultaneous process (Ying et al.). AlexNet is one of the classic convolutional neural networks. AlexNet is deeper than LeNet in terms of network depth. It uses the combined structure of the convolutional layer and pooling layer to obtain features of graphic images. This research mainly explores the decision-making application of the cloud-fog hybrid model based on the improved convolutional neural network in financial services in smart medical care, so as to optimize the financial procedures for admission and discharge through the new model and shorten the patients' wait in line, reduce hospital costs, and improve patient satisfaction.

## 2. Model Introduction

### 2.1. AlexNet Network

As a commonly used convolutional neural network for deep learning [12, 13], AlexNet is improved based on the classic network LeNet, and on this basis, it can obtain more deep image features by extending the depth of the network. AlexNet is deeper than LeNet in terms of network depth and uses the combined structure of the convolution layer and pooling layer to obtain the features of graphic images [14]. At the same time, AlexNet also uses dropout regularization to suppress overfitting and uses the ReLU function instead. The sigmoid function is used as the activation function of the convolutional neural network, and the results prove that the ReLU function performs better in the deep convolutional neural network and also solves the problem of gradient dispersion and gradient disappearance caused by the sigmoid function (A et al., 2021), and the ReLU function has a faster learning speed. AlexNet has a total of 8 layers of network structure. The first 5 convolutional layers include 1 11 × 11 convolutional layer, 1 5 × 5 convolutional layer, and 3 3 × 3 convolutional layers, with 2 maxpool and 3 FC layers.

### 2.2. BN Normalization Algorithm

The role of the BN (batch normalization) layer is to prevent the gradient from dispersing and disappearing [15] so that a larger learning rate can be set when training the network, which significantly improves the training speed of the network model so that the model training does not rely too much on parameter initialization. To some extent, it reduces the dropout layer in the convolutional neural network [16]. So, its importance is the same as other structural layers in the network, and it is also an important structural part of the convolutional neural network. In general, the design of convolutional neural networks is more inclined to place the BN layer after the convolutional layer and the fully connected layer; of course, it can also be placed before the activation function [17]. The principle is that when each layer of the network is input, another normalization layer is inserted, that is, a normalization process is performed first, and then the next layer is entered, and it is a learnable one with parameters (*γ*, *β*) of the network layer. Assuming the input is n-dimensional, the normalization formula is as follows:

(1) $$\begin{array}{c} X=\left(x^{\left(1\right)}\cdots x^{\left(n\right)}\right). \end{array}$$

Normalize each dimension, then

(2) $$\begin{array}{c} x=\frac{x^{\left(1\right)}-E\left[x^{\left(k\right)}\right]}{\sqrt{Var\left[x^{\left(k\right)}\right]}}. \end{array}$$

If you just use the above normalization formula to normalize the output of a certain layer of the network and then send it to the next layer, this will affect the features learned by the output data of the previous layer, so the transformation and reconstruction method is introduced. The idea is to introduce the learnable parameters *γ* and *β*, and the formula is as follows:

(3) $$\begin{array}{c} y^{\left(k\right)}=\gamma^{\left(k\right)}{\hat{x}}^{\left(k\right)}+\beta^{\left(k\right)},\\ \gamma^{\left(k\right)}=\sqrt{Var\left[x^{\left(k\right)}\right]},\\ \beta^{\left(k\right)}=E\left[x^{\left(k\right)}\right]. \end{array}$$

It can be seen from the above formula that by reconstructing the parameters *γ* and *β* and learning these two parameters, the original features learned by a certain layer in the convolutional neural network can be recovered. However, in the actual test, the following formula is still used:

(4) $$\begin{array}{c} \hat{x}=\frac{x-E\left[x\right]}{\sqrt{Var\left[x\right]+\varepsilon }}. \end{array}$$

### 2.3. Cloud Model

Since the concept of cloud computing appeared in 2006, the two IT technologies of computing and network have been continuously integrated and then coexisted with each other, which has effectively promoted the development of the information society [18]. In these IoT scenarios, a more secure, faster, and more stable computing mode is required, and at the same time, computing needs to have better mobility support [19]. The above requirements cannot be met for cloud computing with high latency, low security, and reliability. Therefore, the concept of fog computing emerges as the times require.

Fog computing was proposed by Cisco in 2011. It deploys a large number of micro-fog node data centers with limited computing and storage capacity between the cloud and the object to disperse the computing pressure of the cloud center and reduce the amount of data transmitted to the remote network [20]. Due to the limited computing power of fog computing itself, it cannot replace cloud computing, but expands and supplements it. The integrated use of these two technologies not only retains the powerful computing and storage advantages of the cloud layer but also expands the scope of network computing. At the near-user end, that is, the network edge, network computing has lower latency and higher location awareness [21]. The benefits brought by fog computing have made a huge impact in the IT industry. In 2015, IT industry leaders such as Cisco, Dell, and Intel jointly established the OpenFog Consortium to promote the rapid development of cloud-fog hybrid computing. Today, more than fifty institutions from North America, Asia, and Europe have joined the Open Fog Alliance [22]. In 2018, the National Institute of Standards and Technology restandardized the definition of fog computing on the basis of Cisco's years of fog computing research: fog computing is a combination of smart devices and traditional cloud data centers. A horizontal computing model combines physical and virtual resources. With the standardization of fog computing-related concepts, the technical architecture of cloud-fog hybrid computing has become increasingly mature [23].

#### 2.3.1. Cloud Computing Center Layer

In the cloud-fog hybrid computing model, the traditional cloud computing center is retained. The cloud computing center uses a large number of virtual resources and provides extremely strong computing power and storage capacity with the help of task scheduling, load balancing, and parallel computing technologies to meet the processing of complex computing tasks. In the Internet of Things scenario, the cloud computing center is suitable for intelligent analysis and learning of large data volume information and storage of historical data, which is a supplement to the computing capability of the fog layer.

#### 2.3.2. Network Layer

The network layer includes the access network layer and the core network layer. The access network layer mainly connects end-user equipment and fog layer node equipment through network equipment, which includes both wired and wireless networks. The core network connects the cloud computing center and the fog layer computing nodes through the wired network.

#### 2.3.3. Fog Computing Layer

The introduction of the fog computing layer is the core of cloud-fog hybrid computing, which requires certain business processing and data computing capabilities. At the same time, the fog computing layer also needs to be able to cooperate with the cloud layer to carry out reasonable network control and resource scheduling to complete more complex computing and storage tasks. In addition, the scale of computing nodes in the fog computing layer may also become huge due to business requirements, and the hardware and software costs of a single computing node are relatively low. In order to meet the above functional requirements, in terms of hardware, the fog computing layer can be composed of general-purpose servers, white-label switches, routers, and other devices. In terms of software, in addition to the software system responsible for business computing and processing, it is also necessary to introduce software defined network (SDN) technology responsible for network traffic control and forwarding, and network functions virtualization (NFV) responsible for providing virtual network functions.  Table 1 shows the main software and hardware resources required for the general fog computing layer.

Building fog computing nodes is an important part of fog computing layer construction. The Central Office Rearchitected as a Datacenter (CORD), DC transformation of network computer room, project promoted by the Open Network Alliance (ONF) basically meets the requirements of fog-layer computing nodes. The CORD platform integrates SDN, NFV, and other technologies and provides the possibility of fog-layer computing, traffic control, and network services with the help of hardware resources such as general-purpose servers and white-brand switches. If business services are added to it, it will become a suitable fog layercompute node.

#### 2.3.4. End User Layer

In the era of the Internet of Things, there are more and more types of devices in the end-user layer, including smartphones, computers, smart wearable devices, and various sensors. In order to realize the vision of the Internet of Everything, these intelligent terminal devices are connected together through wired or wireless networks, thus creating the necessity for the development of cloud-fog hybrid computing. In cloud-fog hybrid computing, the intelligent terminal device is the initiator of the task, and the task is forwarded to the corresponding fog computing node after being scheduled by the network device in the access network. After the task is processed by the fog layer and cloud layer, the processing result will be sent back to the terminal device through the network.

## 3. Network Improvements

### 3.1. Improvement Method

In this section, the UCNN network is designed on the basis of AlexNet, and the convolution group structure is introduced into the AlexNet network, that is, the convolution group convset of the small convolution kernel. The advantage of this structure design is that it is convenient to adjust the algorithm, and the convolution group can be directly added [24]. In this convolution group, there is a 1 × 1 convolutional layer at the beginning and the end, which can be connected with convolutional layers of any scale. A 3 × 3 convolution kernel and a 5 × 5 convolution kernel are used in the middle. The structure is shown in Figure 1.

A convolutional neural network is mainly composed of the input layer, convolution layer, activation layer, pooling layer, and fully connected layer. The network model in this paper introduces more than 3 of the above convolution groups to replace the 11 × 11 large convolution kernels in the AlexNet network. Each convolution group introduces 4 3×3 convolution layers and 2 max-pooling layers and then adds a batch normalization layer (BN layer), which can speed up the convergence of the model.The convolutional layers are supplemented with 0 to prevent edge pixels from being omitted when the convolution kernel performs convolution calculations. Using dropout regularization, all neurons are discarded according to the probability of 0.3, which simplifies the entire network model, suppresses overfitting, and further improves the classification ability of the model [25].

Dropout regularization can effectively suppress the phenomenon of overfitting. The main idea is that a part of the neurons in each layer of the network is randomly discarded, and the probability of random discarding is set according to the training situation of the model. This paper has carried out many experiments, starting from the probability of 30%, 40%, and 50%. The experimental results show that the random discarding of neurons with a probability of 0.3 is the best. Therefore, this paper sets the dropout regularization parameter to 30%, which simplifies the network structure while suppressing overfitting.

In this paper, the main idea of improving the AlexNet network structure is to replace the 11 × 11 large convolution kernel with a convolution group of small convolution kernels to extract more subtle features in smart medical financial services, and other convolution layer parameters are set the same. In the overall network structure improvement, convolution groups with small convolution kernels have been introduced 4 times. The two improved methods are given in Table 1. Figures 2 and 3 are the experimental results of the recognition accuracy of the two design methods on the FER2013 and CK+ datasets, respectively.

The results of the cubic and quaternary convolution groups are studied. From Figures 2 and 3, it can be found that the cubic convolution group has higher accuracy than the quaternary convolution group, and the accuracy rate of the quaternary convolution group is higher. In FER2013 and CK+, the two datasets used in this experiment are always slightly lower than the cubic convolution group. In the following fitting, the cubic convolution group is selected.

### 3.2. UCNN Network Structure

Compared with the classification accuracy, the effect of introducing 3 convolution groups is better, so this paper finally adopts the introduction of 3 convolution groups as the final network model, named UCNN (Unit CNN) network.  Figure 4 shows the whole improved network model diagram.

## 4. Simulation Results and Analysis

This section first introduces the dataset used and then performs data enhancement on the dataset. The improved network model in this paper is used to train and test the expression dataset and compared with a variety of newer expression recognition methods; the comparison results show that the improved network model is more effective. The experimental environment of this paper is a Windows system, the deep learning model is Pytorch, the CPU is Intel i59600kf, and the GPU is NVIDIA GTX1080ti.

### 4.1. Dataset Processing

#### 4.1.1. FER2013 Dataset

The FER2013 dataset is a commonly used identification research dataset, which itself has been divided into a training set, validation set, and test set. Among them, there are 28,709 training sets, 3,589 validation sets, and 3,589 test sets.

#### 4.1.2. CK+ Dataset

The CK+ dataset was released in 2010. It is a dataset with a larger amount of data obtained by expanding the dataset on the CK dataset. In this paper, 30% of the dataset is divided into the test set, and 70% is divided into the training set.

### 4.2. Data Augmentation

Convolutional neural networks are often supported by a large number of parameters. Some large neural networks, such as GoogleNet, even have millions of network parameters. To make these huge network parameters work properly, a large amount of data is required. Train the network for a long time. However, the reality is that there is not that much data to work with. Therefore, data augmentation plays a great role in network training. It can expand the amount of data, improve the generalization ability of the model, and improve the robustness of the model. The data augmentation method used in this paper is random sampling.

### 4.3. Improved Analysis

This paper improves the original AlexNet, introduces three convolution groups with small convolution kernels to replace the 11 × 11 convolution kernels in the original AlexNet, constructs a new network UCNN, and uses the UCNN network on the FER2013 dataset and CK+ dataset, respectively. Train and test: the dataset has been expanded, and the CK+ dataset has been expanded to 2000, of which 70% are used as training sets and 30% are used as test sets. The FER dataset is not expanded, because the amount of data in the original dataset itself is relatively large.

Figures 5 and 6 show the training accuracy and test accuracy of the improved network UCNN on the CK+ dataset and the FER2013 dataset. It can be seen that the UCNN network performs well on the two datasets, where the dotted line represents the training accuracy. The solid line represents the test accuracy, which reached the recognition rate of 98% and 68.01% respectively, and there is no obvious overfitting phenomenon, indicating that the network in this paper has a relatively good generalization ability.

On the FER2013 and CK+ datasets, other network models are used for testing, and compared with the UCNN network, the results are shown in Figures 7 and 8.

Reference [26], reference [27], and reference [28] all conducted experiments on the FER2013 dataset, and reference [29], reference [30] and reference [31] all conducted experiments on the CK+ dataset. As can be seen from the chart, the method in this paper performs the best on both datasets.

## 5. Conclusion

The information system compiled according to the internal control requirements objectively enforces and regulates the operation behavior of operators, eliminates arbitrary and subjective factors, and is an important means to reduce the risk of errors and fraud. Aiming at the low utilization rate of small and medium-sized convolutional neural networks in smart medical financial systems, this study designs the UCNN network, which uses the convolution group of small convolution kernels to replace the 11 × 11 large convolution kernels in the AlexNet network. Small convolution kernels help to extract more subtle features of the original data, thereby improving the recognition rate. A BN batch normalization layer is added after each convolution group to prevent the gradient from disappearing and improve the training speed of the network. In order to reduce the network parameters, a fully connected layer in the original structure is removed, and dropout regularization is added behind the remaining two fully connected layers to further prevent overfitting. During the training process, the dataset was enhanced to solve the problem of insufficient data. The research results are as follows: (1) the improved network UCNN based on AlexNet designed in this paper has a simpler structure, fewer parameters, faster model convergence speed, and higher recognition rate compared with the current newer methods; FER2013 and CK+ datasets achieved recognition rates of 98% and 68.01%, respectively; (2) compared with the quadruple convolution group, the cubic convolution group has higher accuracy, and the accuracy of the cubic convolution group is higher than that of the quaternary convolution group by 67.80% and 96.55%; (3) data enhancement significantly expands the data volume, improves the generalization ability of the model, and improves the robustness of the model [32].

## Figures and Tables

**Figure 1:** Structure of convolution group convset.

**Figure 2:** Comparison of two networks on FER2013 dataset.

**Figure 3:** Comparison of two networks on CK+ dataset.

**Figure 4:** UCNN network structure.

**Figure 5:** Training and test performance of the UCNN network on FER2013 dataset.

**Figure 6:** Training and test performance of the UCNN network on CK+ dataset.

**Figure 7:** Comparison of training and test performance of recognition rate between this method and other methods on FER2013 dataset.

**Figure 8:** Comparison of recognition rate between this method and other methods on CK+ dataset.

**Table 1:** Comparison of classification accuracy on FER2013 and CK+ datasets during model improvement.

Ways to improve	Precision	
	Dataset of FER2013	Dataset of CK+
Introduce 4 convolution groups	67.80	96.55

Introduce 3 convolution groups	68.55	97.51

## Data Availability

The dataset used to support the findings of this study is available from the corresponding author upon request.
